# MRI texture analysis in predicting treatment response to neoadjuvant chemoradiotherapy in rectal cancer

**DOI:** 10.18632/oncotarget.23813

**Published:** 2017-12-22

**Authors:** Yankai Meng, Chongda Zhang, Shuangmei Zou, Xinming Zhao, Kai Xu, Hongmei Zhang, Chunwu Zhou

**Affiliations:** ^1^ Department of Radiology, National Cancer Center/Cancer Hospital, Chinese Academy of Medical Sciences and Peking Union Medical College, Beijing, China; ^2^ Department of Pathology, National Cancer Center/Cancer Hospital, Chinese Academy of Medical Sciences and Peking Union Medical College, Beijing, China; ^3^ Department of Radiology, The Affliated Hospital of Xuzhou Medical University, Xuzhou, Jiangsu Province, China

**Keywords:** rectal cancer, texture analysis, magnetic resonance imaging, response assessment, neoadjuvant chemoradiotherapy

## Abstract

To evaluate the importance of MRI texture analysis in prediction and early assessment of treatment response before and early neoadjuvant chemoradiotherapy (nCRT) in patients with locally advanced rectal cancer (LARC). This retrospective study comprised of 59 patients. The tumoral texture parameters were compared between pre- and early nCRT. Area Under receiver operating characteristic (ROC) Curves [AUCs] were used to compare the diagnostic performance of statistically significant difference parameters and logistic regression analysis predicted probabilities for discriminating responders and nonresponders. The Standard Deviation (SD), kurtosis and uniformity were statistically significantly difference between pre- and early nCRT (*p* = 0.0012, 0.0001, and < 0.0001, respectively). In pathological complete response (pCR) group, pre-uniformity and pre-Energy were significantly higher than that of nonresponders (*p* = 0.03 and *p* < 0.01, respectively), while the pre-entropy in nonresponder was reverse (*p* = 0.01). The diagnostic performance of pre-kurtosis and pre-Energy were higher in tumor regression grade (TRG) and pCR group (AUC = 0.67, 0.73, respectively). Logistic regression analysis showed that diagnostic performance for prediction responder and nonresponder did not significantly improve compared with to pre-uniformity, energy and entropy in pCR group (AUC = 0.76, *p* = 0.2794, 0.4222 and 0.3512, respectively). Texture parameters as imaging biomarkers have the potential to prediction and early assessment of tumoral treatment response to neoadjuvant chemoradiotherapy in patients with LARC.

## INTRODUCTION

Neoadjuvant chemoradiotherapy (nCRT) followed by total mesorectal excision (TME) is the recommended standard therapy for patients with locally advanced rectal cancer (LARC) [1–3]. This treatment strategy has improved locoregional control, and rates of sphincter preservation [1, 2] and lead to significant pathologic complete response (pCR) defined as the absence of viable tumor cells after full pathologic examination of the resected specimen (ypT0N0M0) in a significant proportion of patients [4, 5]. In these patients with pCR to nCRT, some investigations have indicated that surgery can be omitted and the non-operative treatment strategy with strict follow-up (watch-and-wait strategy) may be safe and associate with good survival rates [4–7]. Accurate response assessment to nCRT prior to the start and early treatment can enhance clinical care management by enabling the personalization of treatment plans based on predicted outcome.

Magnetic resonance imaging (MRI) have been the most extensively studied response evaluation for nCRT in patients with LARC. Different MRI biomarkers including tumor volume, apparent diffusion coefficient (ADC) values, perfusion parameters of dynamic contrast-enhanced MRI (DCE-MRI), and parameters derived from intravoxel incoherent motion diffusion-weighted imaging (IVIM-DWI) have been investigated [8–11]. But these imaging markers have limitations in predicting treatment response. Tumor volume measurement methodology is not practically feasible owing to the time-consuming nature. The DWI is a functional imaging technique that analyses differences in intracellular and extracellular space random Brownian motion of water protons to discriminate between tissues of varying cellularity. By measuring the ADC values, DWI has shown to be more valuable to monitor tumor response before and after treatment than morphologic MRI, but there is no consensus on the diagnostic accuracy in rectal cancer, the performance varies dramatically ranging from 0.51 to 0.85 [8, 12, 13]. Although studies prove that DCE-MRI and IVIM-DWI modalities are useful in treatment response of rectal cancer, these studies are still in extremely preliminary stages [11, 14].

There is increased interest in the field of radiomics due to the limitations in existing imaging modalities and the concept that radiological images hold more information than that is being utilized. Radiomics is defined as the high throughput extraction of quantitative imaging features or texture parameters from imaging to decode tissue pathology and creating a high dimensional data set for feature extraction [15]. Recently, as a potentially imaging biomarker, assessing tumor heterogeneity in relation to treatment response by extracting textural features has emerged [16–18]. Texture analysis (TA) is a noninvasive method of assessing the intratumoral heterogeneity. To date, there is very little research carried out to assess whether TA of MRI in rectal cancer can potentially be used as an imaging biomarker for early response to nCRT [19, 20]. The first study demonstrated that pre-treatment kurtosis was the best predictor to distinguish pCR from partial response (PR) and nonresponse (NR), and the diagnostic performance was 0.86. However, both studies included some patients with stage T1-2N+M0, and the validation was not performed, particularly in T3-T4 rectal cancer.

The aim of this study was to investigate whether TA of rectal cancer based on T2-weighted MRI can predict and provide an early assessment of tumoral response in patients with LARC treated with nCRT.

## RESULTS

### Patient population

The study cohort consisted of 59 consecutive patients (39 males and 20 females; mean age - 54 years; age range - 46–62 years). According to the reference standards, TRG 1–2, pCR, and T-downstaging were found in 30 (50.8%), 15 (25.4%), and 28 (47.5%) patients, respectively. Baseline characteristics of the patient population and the pathologic findings of the surgical specimen are summarized in Table 1.

**Table 1:** Baseline patient characteristics and histopathological findings

Characteristics	Value
Total patients	59
Age (years)	
≤ 60	42(71.2%)
> 61	17(28.8%)
Primary mass location(from anal verge)	
0–5 cm	27(45.8%)
5.1–10 cm	29(49.2%)
10.1–15 cm	3(5.0%)
pre-nCRT clinical T stage	
T3	37(62.7%)
T4	22(37.3%)
pre-nCRT clinical N stage	
N0	11(18.6%)
N+	48(81.4%)
post nCRT TRG group	
TRG1-2	30(50.8%)
TRG3-5	29(49.2%)
ypT stage	
T0	16(27.1%)
T1	1(1.7%)
T2	11(18.6%)
T3	30(50.9%)
T4	1(1.7%)
ypN stage	
N0	15(25.4%)
N+	44(74.6%)

TRG indicates tumor regression grade; nCRT, neoadjuvant chemoradiotherapy; ypT/N stage, therapy pathological T/N stage.

### Interobserver agreement

There was a moderate-to-excellent interobserver agreement in the histogram and first-order texture metrics, with intraclass correlation coefficients ranging from 0.60 to 0.99. Full results are listed in Table 2.

**Table 2:** ICC of interobserver in TA parameters before and early nCRT

	ICC	95%CI
**pre-nCRT**		
Mean value	0.99	0.99–1.00
SD	0.93	0.89–0.96
skewness	0.79	0.68–0.87
kurtosis	0.86	0.78–0.92
uniformity	0.88	0.81–0.93
Energy	0.97	0.95–0.99
Entropy	0.97	0.95–0.99
**Early nCRT**		
Mean value	0.99	0.99–1.00
SD	0.95	0.92–0.97
skewness	0.7	0.55–0.81
kurtosis	0.6	0.40–0.74
uniformity	0.91	0.86–0.95
Energy	0.96	0.93–0.97
Entropy	0.96	0.93–0.98

ICC indicates intraclass correlation coefficients.

### Differences of TA between pre- and early nCRT

There was a trend for SD and energy to be lower in pre-nCRT than in early nCRT, while Mean value, skewness, kurtosis, uniformity, and entropy reversed. Only SD, kurtosis, and uniformity were significantly different between pre- and early nCRT (*p* = 0.0012, 0.0001, and < 0.0001, respectively) (Figure 1). There was no significant difference in mean value, skewness, Energy, and entropy between pre- and early nCRT.

**Figure 1:** Box-and whisker plot shows SD, kurtosis and uniformity are statistically significantly difference between pre- and early CRT groups

### Responder and nonresponder parameters

The pre-kurtosis was significantly higher in patients with responder vs. nonresponder in TRG group (3.57 vs 3.24, *p* = 0.02). There were significant difference in pre-uniformity (0.82 vs 0.79, *p* = 0.03), pre-energy (0.95 vs 0.50, *p* < 0.01) and pre-entropy (0.22 vs 1.39, *p* = 0.01) between patients with responder and patients with nonresponder in pCR group. Full results are listed in Tables 3–4.

**Table 3:** Comparison of tumor texture analysis parameters between TRG1-2 and TRG3-5 groups

	TRG		
Parameters	TRG1–2(*n* = 30)	TRG3–5(*n* = 29)	*p*
pre-mean value	226.42(165.19–284.39)	239.08(170.24–288.02)	0.50
pre-SD	40.72(32.42–61.49)	47.51(35.76–59.27)	0.40
pre-skewness	0.30(0.10–0.63)	0.22(0.04–0.40)	0.36
pre-kurtosis	3.5734(3.24–4.25)	3.24(2.88–3.69)	0.02
pre-uniformity	0.80(0.78–0.84)	0.79(0.77–0.82)	0.51
pre-energy	0.72(0.45–0.95)	0.49(0.40–0.84)	0.09
pre-entropy	0.88(0.20–1.52)	1.41(0.57–1.61)	0.12
early mean value	207.80(160.10–243.40)	208.80(169.88–310.87)	0.64
early SD	51.97(34.99–65.38)	44.67(36.47–63.98)	1.00
early skewness	0.21(0.01–0.49)	0.23(-0.08–0.35)	0.63
early kurtosis	3.11(2.75–3.55)	2.89(2.62–3.33)	0.16
early uniformity	0.77(0.72–0.81)	0.77(0.73–0.79)	0.89
early energy	0.70(0.52–0.91)	0.68(0.41–0.89)	0.52
early entropy	0.92(0.36–1.33)	1.04(0.45–1.61)	0.51

TRG indicates tumor regression grade. Data are reported as mean (95% Confidence Interval). Significant differences are represented in bold.

**Table 4:** Comparison of tumor texture analysis parameters between pCR and nonpCR groups

	pCR		
Parameters	pCR(*n* = 15)	non pCR(*n* = 44)	*p*
pre-mean value	185.76(165.38–245.85)	239.54(169.17–286.81)	0.26
pre-SD	33.40(28.91–45.49)	49.25(34.81–60.90)	0.06
pre-skewness	0.26(0.11–0.55)	0.24(0.045–0.58)	0.89
pre-kurtosis	3.56(3.39–4.11)	3.40(3.01–3.92)	0.09
pre-uniformity	0.82(0.80–0.84)	0.79(0.76–0.82)	**0.03**
pre-energy	0.95(0.57–0.97)	0.50(0.42–0.87)	**< 0.01**
pre-entropy	0.22(0.14–1.37)	1.39(0.46–1.60)	**0.01**
early mean value	199.50(157.40–224.08)	209.84(169.53–315.32)	0.28
early SD	41.76(32.02–62.64)	53.38(36.61–65.92)	0.26
early skewness	0.17(-0.05–0.42)	0.23(-0.026–0.43)	0.81
early kurtosis	2.96(2.76–3.45)	3.00(2.61–3.43)	0.58
early uniformity	0.78(0.72–0.80)	0.77(0.73–0.80)	0.75
early energy	0.72(0.53–0.93)	0.68(0.45–0.87)	0.22
early entropy	0.88(0.29–1.30)	1.05(0.50–1.58)	0.17

pCR indicates pathological complete response. Data are reported as mean (95% Confidence Interval). Significant differences are represented in bold.

### Diagnostic performance

The AUC to discriminate patients with responder from patients with nonresponder were 0.67 for pre-kurtosis in TRG group. This allowed a prediction of response with a sensitivity of 55.17% and a specificity of 73.33% at an optimal cutoff value of ≤ 3.29. For the pre-uniformity, pre-energy and pre-entropy in pCR group, ROC curve analysis showed an AUC of 0.69, 0.73 and 0.72 at an optimal cutoff value of ≤ 0.79, ≤ 0.93 and > 0.22, respectively. This allowed for a prediction of response with a sensitivity of 54.55, 84.09, 86.36% and a specificity of 93.33, 53.33, 53.33%, respectively. The logistic regression analysis for the combined parameters (pre-uniformity, pre-energy, and pre-entropy) achieved an AUC of 0.76 (cutoff value > 0.64, SE 79.55%, SP 66.67%) in pCR group. This was not a significant improvement compared with the pre-uniformity, pre-energy and pre-entropy in pCR group (*p* = 0.2794, 0.4222 and 0.3512, respectively). Full results are listed in Table 5 and Figure 2.

**Table 5:** The predictive values for response according to the different reference standards

Parameters	Cut-off value	AUC (95% CI)	Sensitivity (%)	Specificity (%)
**TRG**				
pre-kurtosis	≤ 3.29	**0.67(0.54-0.79)**	55.17	73.33
**pCR**				
pre-uniformity	≤ 0.79	0.69(0.55-0.80)	54.55	93.33
pre-energy	≤ 0.93	**0.73(0.60-0.84)**	84.09	53.33
pre-entropy	> 0.22	0.72(0.58-0.83)	86.36	53.33
LOGREGR_Pred1	> 0.64	**0.76(0.63-0.86)**	79.55	66.67

LOGREGR_Pred1 indicate predicted the probability for the combined parameters (pre-uniformity, energy, and entropy) in pCR group. The best AUCs of every subgroup are represented in bold.

**Figure 2:** ROC curves are shown analyzing the discriminatory power of TA parameters and variable derived by logistic regression analysis to distinguish between responder and nonresponder in TRG and pCR groups LOGREGR_Pred1 indicate predicted probability in pCR group. The corresponding AUCs are listed in Table 5.

## DISCUSSION

In this study, we demonstrated the reliable use of TA parameters extracted from conventional T2WI for prediction and early assessment of treatment response of LARC to nRCT according to two different pathological reference standards.

Our results showed that most of the texture parameters (mean value, skewness, kurtosis, uniformity and energy) decreased at the third of week of CRT, with the exception of SD and entropy. In particular, the mean pre-kurtosis in TRG group, pre-uniformity, and pre-energy in pCR group significantly higher in responders compared with nonresponders. While the pre-entropy of pCR group was statistically lower than that of the nonresponder group. The AUCs of pre-kurtosis in TRG group and predicted probabilities derived by logistic regression analysis in pCR group were 0.67 and 0.76, respectively.

Kurtosis reflects peakedness and tailedness of the histogram; it is related inversely to the number of features highlighted [21]. De Cecco et al. research on the correlation of DWI, DCE-MRI and TA parameters indicated that there was a significant negative correlation between kurtosis and ADC [20]. This correlation may be interpreted as a trend that kurtosis was to be higher in pre-CRT than in early CRT.

A preliminary study has recently demonstrated the importance of MRI TA parameters in predicting treatment response of rectal cancer to nCRT [19]. Based on Dworak tumor regression grade, the study demonstrated that kurtosis was the best predictor of tumor response. Pre-kurtosis with medium filtration was significantly lower in patients with pCR in comparison with those with partial response (PR) + nonresponse (NR). Pretreatment AUC for kurtosis using the best medium texture to discriminate between pCR and PR + NR was 0.907. Our results did not correspond well with the results of De Cecco et al. [19]. We speculated that the reasons were due to different patients inclusion criteria and pathologic classification criteria. Our study included only patients with clinical stage T3-4N0/+M0, while patients with stages II (cT3-4N0M0) and III (cT1-4N+M0) were enrolled in the study by De Cecco et al. Contrary to the De Cecco et al. study, our research was based on Mandard tumor regression grade, rather than Dworak criteria [22, 23].

In our study, logistic regression analysis was used to predict probabilities for analyzation. The AUC of predicted probabilities derived by logistic regression analysis before nCRT in pCR group was more favorable than other imaging markers used in previous investigations, in which the prediction of pCR showed moderate accuracy (AUC range, 0.55–0.67) [8, 24]. The TA parameters extraction from MRI hold more information and generated meaningful data than existing imaging modalities to prediction response before nCRT.

There were some limitations to our study. First, this retrospective analysis was not validated by other centers. Further, a prospective investigation with a larger patient database is necessary to ascertain the diagnostic performance of TA parameters to nCRT. Moreover, tumor delineation was performed using a single slice method. The multislice delineation of the tumor area is representative of the whole tumor, but the multislice method is not clinically feasible owing to the time-consuming nature. And, according to Ng, et al. [25], a large cross-sectional area of the tumor is sufficiently represented and provides comparable results to whole tumor analysis. Third, in this study, comparison with the different imaging markers was not made. Finding the optimal imaging marker is essential to ensure sufficiently predictive accuracy. A comprehensive imaging model analyzing the combined efficacy would be needed to assess their combination on the prediction of treatment response. Lastly, we did not perform investigations on the correlation of TA parameters with the corresponding histopathology.

In conclusion, our preliminary study indicates that TA based on T2WI holds promise to prediction and early assessment response and nonresponse to nCRT in patients withLARC.

## MATERIALS AND METHODS

### Study population

This retrospective study was approved by the Medical Ethics Committee of National Cancer Center/Cancer Hospital, Chinese Academy of Medical Sciences and Peking Union Medical College. Informed consents were obtained from all participants. This study was carried out in accordance with the Declaration of Helsinki. The methods were carried out in accordance with the approved guidelines.

From October 2010 to December 2013, all histologically proven locally advanced rectal adenocarcinoma (≥ T3 or lymph node positive) originating within 15 cm of the anal verge and treated with nCRT before TME at our institution were enrolled in this study. The MRI of the pelvis, computed tomography scans of the chest, abdomen, and pelvis were performed as pre-nCRT tumor staging. The exclusion criteria included the history of other malignant tumor, previous pelvic radiotherapy, or contraindication to MRI examination, insufficient quality to analysis.

### Study protocol

All patients underwent MR examinations thrice. The first MR examination (pre-nCRT MRI) was performed for tumor staging before treatment, and the second one (early nCRT MRI, 10-15 fractions after initiation) was used to assess early treatment response at the third week of CRT. The third MRI examination was performed 4-6 weeks after nCRT to monitor the response to treatment. Between 6 and 8 weeks after the nCRT, TME was performed and the gross specimen was analyzed by a dedicated gastrointestinal (GI) pathologist. As our study aimed at prediction and early assessment tumoral treatment response to neoadjuvant chemoradiotherapy, we focused the analyses on pre- and early MR examinations.

### MRI data acquisitions

All MR imaging were performed using a 3T scanner (Signa HDx, General Electrics, Milwaukee, WI, USA) by using a phased-array body coil. A routine clinical imaging protocol was performed including small field of view (FOV) (16 cm×16 cm) high-resolution two-dimensional T2-weighted spin-echo (SE) sequence (repetition time msec/echo time msec, 5160/151; flip angle, 90°; echo train length, 19; slice thickness, 3 mm; matrix, 512 × 512) acquired in three directions, sagittal, oblique coronal (parallel to the long axis of the rectum), oblique axial (perpendicular to the long axis of the tumor), respectively. After that, axial SE DWI echo-planar imaging sequence with background body signal suppression was acquired at b values of 0, 800 sec/mm^2^ (repetition time msec/echo time msec - 4925/68; Nex - 4; slice thickness - 4 mm; matrix - 128×128). Subsequently, axial three-dimensional LAVA DCE-MRI images were acquired. However, only the oblique axial T2-weighted sequence was used for analysis. Patients underwent bowel preparation with antispasmodic medication before the MRI examinations. All these sequences were obtained during free breathing. The average time interval between two MR examinations (the first and the second) and initiation of nCRT were 13 ± 7 days (range, 1-29 days) and 15 ± 2 days (range, 13–21 days), respectively.

### Imaging segmentation and textural features calculation

The Omni-Kinetics software (v. 2.06, GE Healthcare) was used to obtain first order and histogram texture metrics, including mean value, SD, skewness, kurtosis, uniformity, energy, and entropy. One GI radiologist (15 years of experience in interpreting rectal MR images) reviewed the images of all patients on a local picture archiving and communication system (PACS; v. 3.1.S08.1, 2006 Carestream Corporation), then the largest tumor area depicted on the oblique axial T2WI MRI images were chosen to analyze. Pre- and early nCRT MRI images were randomly analyzed by two GI radiologists (10 and 2 years of experience in interpreting rectal MR images, respectively) who were blinded to each other’s results, the clinical and histopathological data related to tumoral treatment response. Regions of interest (ROI) were drawn manually on the selected section of the largest tumor area. The entire area of tumor was included within the ROI, including any viable tumor. The corresponding oblique axial T2WI, DWI, and DCE-MRI imaging were at the readers’ disposal as a reference. Then the pre- and early nCRT texture parameters values were calculated automatically. To remove the MRI noise and improve the parameters reliability, voxel intensities were therefore resampled into equally spaced bins in our study. This discretization step not only reduces image noise, but also normalizes intensities across all patients, allowing for a direct comparison of all calculated textural features between patients.

In this study we explore a feature-based approach to extract and quantify meaningful and reliable information from MR images. In this section we describe in detail the imaging traits assessed in our study, that were used to derive textural features. First-order and histogram statistics describe the distribution of voxel intensities within the MR image through commonly used and basic metrics. Let denote the three dimensional image matrix with voxels and the first order histogram divided by discrete intensity levels. The following first-order and histogram statistics were extracted:

### 1.1 Mean value:

$$\mathrm{mean}=\frac{1}{N}\sum_{i}^{N}X\left(i\right)$$

### 1.2 Standard deviation:

$$\mathrm{standard}\;\mathrm{deviation}={\left(\frac{1}{N-1}\sum_{i=1}^{N}{\left(X\left(i\right)-\bar{X}\right)}^{2}\right)}^{1/2}$$

where $\bar{X}$ is the mean of *X*.

### 1.3 Skewness:

$$\mathrm{skewness}=\frac{\frac{1}{N}\sum_{i=1}^{N}{\left(X\left(i\right)-\bar{X}\right)}^{3}}{{\left(\sqrt{\frac{1}{N}\sum_{i=1}^{N}{\left(X\left(i\right)-\bar{X}\right)}^{2}}\right)}^{3}}$$

where $\bar{X}$ is the mean of *X*.

### 1.4 Kurtosis:

$$\mathrm{kurtosis}=\frac{\frac{1}{N}\sum_{i=1}^{N}{\left(X\left(i\right)-\bar{X}\right)}^{4}}{{\left(\sqrt{\frac{1}{N}\sum_{i=1}^{N}{\left(X\left(i\right)-\bar{X}\right)}^{2}}\right)}^{2}}$$

where $\bar{X}$ is the mean of *X*.

### 1.5 Uniformity:

$$\mathrm{uniformity}=\sum_{i=1}^{N_{i}}P{\left(i\right)}^{2}$$

### 1.6 Energy:

$$\mathrm{energy}=\sum_{i}^{N}X{\left(i\right)}^{2}$$

### 1.7 Entropy:

$$\mathrm{entropy}=-\sum_{i=1}^{N}P\left(i\right)\mathrm{lo}g_{2}\;P\left(i\right)$$

The mean value of the absolute deviations of all voxel intensities around the mean intensity value. The standard deviation is measures of the histogram dispersion, that is, a measure of how much the gray levels differ from the mean. The skewness and kurtosis are the most frequently used central moments. The skewness measures the degree of histogram asymmetry around the mean, and kurtosis is a measure of the histogram sharpness. As measures of histogram randomness we computed the uniformity and entropy of the image histogram.

### Neoadjuvant chemoradiotherapy

All patients were treated with a long course of radiation therapy (RT) at a dose of 50 Gy (in 25 daily fractions of 2 Gy given in 5 weeks) to the whole pelvis. Chemotherapy consisted of oxaliplatin infusion 50 mg/m^2^ on the first day of each week of RT and oral 5-FU derivate capecitabine, 1650 mg/m^2^ bid from the first day to the end of nCRT. Dose reduction of oxaliplatin and capecitabine was not planned.

### Surgical approach

All patients underwent the standard procedure of TME surgery by experienced colorectal surgeons specialized in colorectal oncology [26]. The approach of surgery was chosen by the surgeon based on the different tumor location and results of post nCRT restaging MRI.

### Reference standards of treatment response

The resected specimens were processed and evaluated by a single pathologist (15 years of experience in interpreting rectal cancer pathology) who was not aware of the clinical and MRI findings. Two different pathological reference standards were used to assess tumor treatment response. Resected specimens were examined according to the Union for International Cancer Control (UICC)/American Joint Committee on Cancer (AJCC) TNM system. The tumor regression grade (TRG) was assessed according to Mandard et al. [23]. TRG 1 (complete regression) means the absence of histologically identifiable residual cancer and fibrosis extending through the wall, with or without granuloma. TRG 2 is characterized by the presence of rare residual cancer cells scattered throughout the fibrosis. TRG 3 corresponds to an increase in the number of residual cancer cells, but fibrosis still predominates. TRG 4 indicates residual cancer outgrowing fibrosis. TRG 5 is the absence of regressive changes. Patients with a TRG 1 or 2 were considered as responders, whereas the remaining patients (TRG 3, 4, or 5) were classified as nonresponders. Pathological complete response (pCR) was defined as the absence of any residual tumor cells detected in the surgical specimens (ypT0N0). Patients with ypT0N0 were divided into responder group, while the patients without ypT0N0 were classified into nonresponder group.

### Statistical analysis

Interobserver agreement was characterized by using the intraclass correlation coefficient (ICC) for continuous variables (0–0.20, poor agreement; 0.21–0.40, fair agreement; 0.41–0.60, moderate agreement; 0.61–0.80, good agreement; and 0.81–1.00, excellent agreement). First-order texture parameters (mean value, SD) and Histogram texture parameters (skewness, kurtosis, uniformity, energy, and entropy) were compared between pre- and early nCRT in terms of averages using Wilcoxon signed-rank test. Responder and nonresponder groups were analyzed using the Mann-Whitney test. We used backward method in logistic regression analysis. The TA parameters were selected for multivariable analysis when *p* < 0.05. The predicted probabilities derived by logistic regression analysis for the combined TA parameters were analyzed as variables. Receiver Operating Characteristic (ROC) curves were computed, and corresponding Area Under ROC Curves (AUCs) was calculated to compare the diagnostic performance of statistically significant difference parameters and logistic regression analysis predicted probabilities for discriminating responders and nonresponders. Sensitivity, specificity and cut-off value were performed. Mean values were used for analysis. A *p* value < 0.05 was considered significant for all tests. Statistical analyses were performed with MedCalc software (v. 15.2, Mariakerke, Belgium).

## References

[1] Sauer R, Becker H, Hohenberger W, Rödel C, Wittekind C, Fietkau R, Martus P, Tschmelitsch J, Hager E, Hess CF, Karstens JH, Liersch T, Schmidberger H (2004). Preoperative versus Postoperative Chemoradiotherapy for Rectal Cancer. New England Journal of Medicine.

[2] Bosset JF, Collette L, Calais G, Mineur L, Maingon P, Radosevic-Jelic L, Daban A, Bardet E, Beny A, Ollier JC (2006). Chemotherapy with Preoperative Radiotherapy in Rectal Cancer. New England Journal of Medicine.

[3] van Gijn W, Marijnen CAM, Nagtegaal ID, Kranenbarg EMK, Putter H, Wiggers T, Rutten HJT, Påhlman L, Glimelius B, van de Velde CJH (2011). Preoperative radiotherapy combined with total mesorectal excision for resectable rectal cancer: 12-year follow-up of the multicentre, randomised controlled TME trial. The Lancet Oncology.

[4] Habr-Gama A, Perez RO, Nadalin W, Sabbaga J, Ribeiro U, Sousa AH, Campos FG, Kiss DR, Gama-Rodrigues J (2004). Operative versus nonoperative treatment for stage 0 distal rectal cancer following chemoradiation therapy - Long-term results. Annals of Surgery.

[5] Habrgama A, Perez R, Proscurshim I, Campos F, Nadalin W, Kiss D, Gamarodrigues J (2006). Patterns of Failure and Survival for Nonoperative Treatment of Stage c0 Distal Rectal Cancer Following Neoadjuvant Chemoradiation Therapy. Journal of Gastrointestinal Surgery.

[6] Maas M, Beets-Tan RG, Lambregts DM, Lammering G, Nelemans PJ, Engelen SM, van Dam RM, Jansen RL, Sosef M, Leijtens JW, Hulsewe KW, Buijsen J, Beets GL (2011). Wait-and-see policy for clinical complete responders after chemoradiation for rectal cancer. J Clin Oncol.

[7] Appelt AL, Pløen J, Harling H, Jensen FS, Jensen LH, Jørgensen JCR, Lindebjerg J, Rafaelsen SR, Jakobsen A (2015). High-dose chemoradiotherapy and watchful waiting for distal rectal cancer: a prospective observational study. The Lancet Oncology.

[8] Curvo-Semedo L, Lambregts DM, Maas M, Thywissen T, Mehsen RT, Lammering G, Beets GL, Caseiro-Alves F, Beets-Tan RG (2011). Rectal cancer: assessment of complete response to preoperative combined radiation therapy with chemotherapy--conventional MR volumetry versus diffusion-weighted MR imaging. Radiology.

[9] Ha HI, Kim AY, Yu CS, Park SH, Ha HK (2013). Locally advanced rectal cancer: diffusion-weighted MR tumour volumetry and the apparent diffusion coefficient for evaluating complete remission after preoperative chemoradiation therapy. Eur Radiol.

[10] Intven M, Reerink O, Philippens ME (2015). Dynamic contrast enhanced MR imaging for rectal cancer response assessment after neo-adjuvant chemoradiation. J Magn Reson Imaging.

[11] Nougaret S, Vargas HA, Lakhman Y, Sudre R, Do RKG, Bibeau F, Azria D, Assenat E, Molinari N, Pierredon MA, Rouanet P, Guiu B (2016). Intravoxel Incoherent Motion–derived Histogram Metrics for Assessment of Response after Combined Chemotherapy and Radiation Therapy in Rectal Cancer: Initial Experience and Comparison between Single-Section and Volumetric Analyses. Radiology.

[12] Kim SH, Lee JM, Hong SH, Kim GH, Lee JY, Han JK, Choi BI (2009). Locally advanced rectal cancer: added value of diffusion-weighted MR imaging in the evaluation of tumor response to neoadjuvant chemo- and radiation therapy. Radiology.

[13] Cai PQ, Wu YP, An X, Qiu X, Kong LH, Liu GC, Xie CM, Pan ZZ, Wu PH, Ding PR (2014). Simple measurements on diffusion-weighted MR imaging for assessment of complete response to neoadjuvant chemoradiotherapy in locally advanced rectal cancer. Eur Radiol.

[14] Reyngold M, Niland J, ter Veer A, Milne D, Bekaii-Saab T, Cohen SJ, Lai L, Schrag D, Skibber JM, Small W, Weiser M, Wilkinson N, Goodman KA (2014). Neoadjuvant Radiotherapy Use in Locally Advanced Rectal Cancer at NCCN Member Institutions. Journal of the National Comprehensive Cancer Network.

[15] Gillies RJ, Kinahan PE, Hricak H (2016). Radiomics: Images Are More than Pictures, They Are Data. Radiology.

[16] Ahmed A, Gibbs P, Pickles M, Turnbull L (2013). Texture analysis in assessment and prediction of chemotherapy response in breast cancer. Journal of Magnetic Resonance Imaging.

[17] Brynolfsson P, Nilsson D, Henriksson R, Hauksson J, Karlsson M, Garpebring A, Birgander R, Trygg J, Nyholm T, Asklund T (2014). ADC texture-An imaging biomarker for high-grade glioma?. Medical Physics.

[18] Wang C, Subashi E, Yin FF, Chang Z (2016). Dynamic fractal signature dissimilarity analysis for therapeutic response assessment using dynamic contrast-enhanced MRI. Medical Physics.

[19] De Cecco CN, Ganeshan B, Ciolina M, Rengo M, Meinel FG, Musio D, De Felice F, Raffetto N, Tombolini V, Laghi A (2015). Texture Analysis as Imaging Biomarker of Tumoral Response to Neoadjuvant Chemoradiotherapy in Rectal Cancer Patients Studied with 3-T Magnetic Resonance. Investigative Radiology.

[20] De Cecco CN, Ciolina M, Caruso D, Rengo M, Ganeshan B, Meinel FG, Musio D, De Felice F, Tombolini V, Laghi A (2016). Performance of diffusion-weighted imaging, perfusion imaging, and texture analysis in predicting tumoral response to neoadjuvant chemoradiotherapy in rectal cancer patients studied with 3T MR: initial experience. Abdominal Radiology.

[21] Alobaidli S, McQuaid S, South C, Prakash V, Evans P, Nisbet A (2014). The role of texture analysis in imaging as an outcome predictor and potential tool in radiotherapy treatment planning. Br J Radiol.

[22] Dworak O, Keilholz L, Hoffmann A (1997). Pathological features of rectal cancer after preoperative radiochemotherapy. Int J Colorectal Dis.

[23] Mandard AM, Dalibard F, Mandard JC, Marnay J, Henry-Amar M, Petiot JF, Roussel A, Jacob JH, Segol P, Samama G, Ollivier JM, Bonvalot S, Gignoux S (1994). Pathologic assessment of tumor regression after preoperative chemoradiotherapy of esophageal carcinoma. Clinicopathologic correlations. Cancer.

[24] Generali D, Chen YG, Chen MQ, Guo YY, Li SC, Wu JX, Xu BH (2016). Apparent Diffusion Coefficient Predicts Pathology Complete Response of Rectal Cancer Treated with Neoadjuvant Chemoradiotherapy. Plos One.

[25] Ng F, Kozarski R, Ganeshan B, Goh V (2013). Assessment of tumor heterogeneity by CT texture analysis: can the largest cross-sectional area be used as an alternative to whole tumor analysis?. Eur J Radiol.

[26] Heald RJ, Ryall RDH (1986). Recurrence and Survival after Total Mesorectal Excision for Rectal Cancer. The Lancet.

